# Feasibility and efficacy of a remote real-time wireless ECG monitoring and stimulation system for management of ventricular arrhythmia in rabbits with myocardial infarction

**DOI:** 10.3892/etm.2014.1693

**Published:** 2014-04-25

**Authors:** ZHI-WEN ZHOU, KAI GOU, ZHANG-YUAN LUO, WEI LI, WEN-ZAN ZHANG, YI-GANG LI

**Affiliations:** 1 Department of Cardiology, Xinhua Hospital Affiliated to Shanghai Jiao Tong University School of Medicine, Shanghai 200092, P.R. China; 2 Genix Biotek Science Technology (Shanghai) Co., Ltd., Shanghai 200235, P.R. China

**Keywords:** implantable electronic cardiovascular device, remote, ventricular arrhythmia, management, wireless

## Abstract

The purpose of this study was to explore the feasibility of continuous remote monitoring, and the induction and termination of malignant ventricular arrhythmias (VAs) by a novel implantable electronic cardiovascular device (IECD) system in rabbits with myocardial infarction (MI). The IECD was implanted and MI was induced by ligation of the left anterior descending coronary artery in 20 adult rabbits. Internet-based remote electrocardiogram (ECG) monitoring and ventricular stimulation were conducted in remote locations with internet access. The voltage amplitudes of the stimulation signals were recorded synchronously by remote and surface ECG. Programmed stimulation with regular stimuli and regular stimuli with an added extra stimulus were performed prior to and following the MI surgery to induce and terminate VAs. IECD implantation and MI surgery, as well as qualified remote and bidirectional signal communications between the implanted IECD and extracorporeal system, were successfully achieved in 18 rabbits. The voltage of the stimulation signals recorded by the remote and surface ECGs showed a good correlation with the stimulation current (remote ECG, r=0.972 and surface ECG, r=0.988; P<0.001). Sustained ventricular tachycardia (VT) was induced in five rabbits (5/20, 25%) prior to MI induction and in 12 rabbits (12/16, 75%) following MI induction. Of the 17 induced VTs, 16 were successfully terminated by remote ventricular stimulation. The novel IECD system provides qualified remote wireless ECG monitoring and possesses the potential to induce and terminate VAs by remote ventricular pacing in this rabbit model of MI. Thus, this model of MI may be used to test the efficacy of novel drugs and devices for the management of VAs.

## Introduction

Malignant ventricular arrhythmias (VAs) are the most common cause of sudden cardiac death (1). Arrhythmia monitoring is not available in the majority of patients with VAs, and patients with malignant VAs often are not able to benefit from effective and timely hospital treatment as the majority of VAs occur outside hospital (1,2). Ideally, patients at a high risk of VAs should be continuously monitored to benefit from rapid diagnosis and timely intervention to save lives. Devices that monitor electrocardiograms (ECGs) and provide timely intervention are required to save the lives of patients with malignant VAs (1–4).

Currently available non-invasive techniques, including Holter and ECG telemetry systems, as well as invasive implantable subcutaneous cardiac monitors, are valuable in the detection of arrhythmias, including VAs (1,4–6). Implantable cardioverter-defibrillators (ICDs) detect and terminate VAs and save the lives of patients (7,8). However, false alarms may occur and patients may thus suffer inappropriate shocks (7–10). An ICD with a remote monitoring function has been successfully used to effectively terminate VAs by anti-tachycardia pacing (ATP) and shocks, and manages alarm messages from patients (9–11). The PainFREE Rx and PainFREE Rx II trials showed that ATP terminates the majority of malignant ventricular tachycardias (VTs) (11,12). Animal models are helpful for testing the efficacy of novel drugs and the feasibility of using novel implantable electronic cardiovascular devices (IECDs) with telecommunications technologies for monitoring and terminating VAs.

In the present study, the feasibility of using a novel IECD system with remote wireless cardiac arrhythmia monitoring and ATP functions was explored in rabbits with experimental myocardial infarction (MI).

## Materials and methods

### IECD system

The IECD system was provided by Genix Biotek Science Technology (Shanghai) Co., Ltd. (Shanghai, China). The IECD consists of one electronic component box, <5 ml in volume and 15 g in weight, two ECG monitoring electrodes and one bipolar stimulation electrode (5076 lead; Medtronic, Inc., Minneapolis, MN, USA; Fig. 1). The extracorporeal system consisted of a signal transmit-receive box which connected with the internet or the third-generation communication system (virtual private network system), and a personal computer with ECG monitoring and electrical stimulation software (Fig. 2). The personal computer was also used as a central workstation in the system. The computer received remote digital signals and converted them into real-time ECG data. The real-time ECG was saved as a compressed ECG signal file with precise time stamps for off-line analysis. When the IECD was implanted, the extracorporeal system also remotely sent out a stimulation signal wirelessly to the IECD to stimulate the heart via a stimulation electrode. Two stimulation modes were designed in this IECD system: The regular stimuli (S1S1), and the regular stimuli with an added extra stimulus (S1S2). The stimulation parameters of this IECD system were as follows: Stimulation current between 0.1 and 5 mA, stimulation time length between 0.5 and 5 msec, and stimulation rate between 1 and 50 Hz. In the S1S2 program, every seventh S1 was followed by one S2, and the stimulation interval was 1–10 sec.

### Ethics statement and animal model preparation

A total of 20 adult New Zealand white rabbits (weight, 2.5–3.5 kg; Shanghai Jiagan biological technology Co., Ltd., Shanghai, China) were used. Animal care and handling procedures were approved by the Animal Care and Use Committee, Research Institute of Medicine, Shanghai Jiao Tong University, in accordance with the Guide for the Care and Use of Laboratory Animals published by the National Institute of Health (1996). All animals involved received humane care in compliance with Chinese Association for Accreditation of Laboratory Animal Care. Each surgery was performed under general anesthesia, and all efforts were made to minimize suffering.

The rabbits were anesthetized with sodium pentobarbital (30 mg/kg induction, and 2.0–5.0 mg/kg/h with intermittent boluses as required). The skin was excised at the location of the jugular vein, and then the jugular vein was separated. The monitoring electrodes of the IECD were fixed subcutaneously, with one electrode at the right upper limb joint as the cathode and another at the left upper quadrant of the abdomen as the anode. Following the incision of the jugular vein, the stimulation electrode of the IECD was implanted in the right ventricle through the jugular vein aided by laboratory digital subtraction angiography (Fig. 2). Following confirmation of the lowest stimulation current threshold (0.2–1.0 mA) of ventricle pacing, the stimulation electrode was fixed and the IECD was implanted subcutaneously into the back of each rabbit, close to the cervicum. After the IECD was implanted, a left thoracotomy was performed through the fourth intercostal space to expose the heart. The major branch of the left anterior descending branch was occluded to induce MI. The rabbits with the implanted IECD were placed within 10 m of the signal transmit-receive box. To prevent infections, 400,000 U penicillium sodium were injected intramuscularly daily for 3–5 days as required.

### Remote ECG monitoring and ventricular stimulation protocol

The cardiac electrical signal filtration used for the ECG was between 0.5 and 100 Hz. The rabbits with the implanted IECD were placed at different distances from the signal transmit-receive box to test the quality of the wireless ECG signal and the intensity of the stimulating signals. The wireless signal intensity of the IECD implanted in the rabbits was also checked with a home-made electronic detection device, based on low power consumption and wireless transceiver technologies (CC1101; Texas Instruments Inc., Dallas, TX, USA) and upper monitor control software. The signal-to-noise ratio (SNR) was used to analyze the IECD wireless signal intensity, which was deemed reliable if the SNR was >80 decibels (dB), according to the CC1101 manufacturer’s instructions (13).

Prior to and on the second day following the MI surgery, the surface ECG leads were connected with the cathode and anode electrodes, which were placed near the monitoring electrodes of the IECD in the animal laboratory. In a remote location with internet access, another investigator from the group manipulated the internet-based remote system using a personal computer for remote ECG monitoring and ventricular stimulation. Surface and remote ECG data were recorded synchronously, and the voltage amplitudes of the stimulation signal with different stimulating currents were compared subsequently. Simultaneously, the time delay between the beginning of the stimulation command at the remote personal computer and the appearance of stimulation signals on the ECG was tested. Sustained VT was defined as VT continuing for >30 sec. The remote S1S1 and S1S2 stimulation programs were repeated to induce VT, and then to terminate the sustained VT. Briefly, the initial S1S1 stimulation rate, which was >20% of the sinus rhythm with 10 msec descending steps, was used until a refractory period appeared. The initial S1S2 stimulation rate, which was >20% of the sinus rhythm with 10 msec S1 descending steps and 5 msec descending S2 steps, was also used until a refractory period appeared. The S1S1 and S1S2 stimulation programs were repeated 7–10 times for each electrophysiological study, or until sustained VT and/or ventricular fibrillation (VF) appeared. If sustained VT was induced, ventricular pacing with a rate >20% of the induced VT rate was performed routinely to terminate it. If VF was induced, S1S1 and S1S2 ventricular stimulation was attempted to terminate the VF. We checked the function of monitoring/stimulation everyday to observe the IECD battery capacities by using the 2 rabbits until the battery was exhausted.

### Statistical analysis

All data are expressed as the mean ± standard deviation. Linear regression analysis was used to determine the correlation among the stimulation current and the amplitude of the stimulation voltage signal shown by the surface and remote ECGs. P<0.05 was considered to indicate a statistically significant difference.

## Results

### Animals

Two out of the 20 rabbits died from hemorrhages during the MI surgery. The IECD implantation and MI induction were successful in the remaining 18 rabbits. Two rabbits died of spontaneous VT/VF and cardiac arrest within 24 h after the surgery, and another rabbit died of induced VT/VF during S1S1 and S1S2 stimulation on the second day after the surgery. A total of 13 rabbits were sacrificed with deep anesthesia within one week after the induction of MI. Remote wireless ECG monitoring and stimulation function were conducted in the remaining two rabbits for three months to observe the battery capacities of the IECD.

### Remote wireless ECG monitoring and ventricular stimulation

The SNR was between −40±5.2 dB at 1 m and −61±3.8 dB at 10 m, demonstrating that the wireless signal intensity of the implanted IECD was stable and reliable within a 10-m distance. The ECG monitoring and ventricular stimulation were successfully performed within 10-m distances. The system achieved real-time ECG monitoring with a 2–3-sec time delay depending on network speed, and the ECG signal was saved in a compressed file with precise time stamps. The morphology of the remote ECG signal was similar to that of the surface ECG signal (Fig. 3).

S1S1 and S1S2 stimulations were performed successfully in 16 rabbits on the second day following the MI surgery (Fig. 4). The stimulation signal voltage recorded by the surface and remote ECGs increased in proportion with the increasing stimulation current (remote ECG, r=0.972 and surface ECG, r=0.988; P<0.001), and the voltage of the stimulation signals recorded by the remote ECG also correlated well with those of the surface ECG (r=0.960; P<0.001; Fig. 5).

The compressed ECG signal file of those 16 rabbits was analyzed offline. Within one week after the MI induction, spontaneous VTs were identified in six rabbits, including three with sustained VTs. Two of the six rabbits died due to spontaneous VT/VF and cardiac arrest within 24 h after the MI induction and the other spontaneous VT was self-terminated.

### Induction and termination of VAs and battery capacities

Sixteen rabbits were stimulated remotely by S1S1 and S1S2 to induce VT and then terminate it afterwards. Sustained VT was induced in five rabbits prior to the MI surgery (5/20, 25%) and terminated successfully. Following the MI surgery, sustained VT was induced in 12 rabbits (12/16, 75%), and four of these VTs deteriorated into VF. The induced sustained VTs/VF were terminated successfully in 11 of the 12 rabbits by S1S1 and S1S2 ventricular stimulation and failed in one, which died of induced VT/VF. Three of the induced VFs were also terminated successfully by ventricular stimulation (Fig. 6). Overall, of 17 induced VTs, 16 (94%) were successfully terminated. The system continued to work well with prolonged use, and high-fidelity and stable wireless ECG signaling was observed for three months in the two rabbits used for observing the battery capacities.

## Discussion

The present study is the first report concerning the feasibility of this novel IECD system in terms of remote monitoring, and the induction and termination of VAs in a rabbit model of MI, to the best of our knowledge. The results show that this novel IECD system monitors, induces and terminates VAs in rabbits with MI. Thus, this model of MI may be useful in studies on novel drugs and devices for the management of VAs.

In the present study, real-time remote wireless and bidirectional signal communication between the IECD implanted in rabbits with MI and the extracorporeal system was achieved effectively and satisfactorily. The remote ECG was able to identify P waves, QRS complexes, T waves and arrhythmias, and to detect VTs and VF correctly. High-fidelity and stable wireless ECG signaling was observed at a remote workstation for three months. Real-time and continuous ECG was saved as a compressed ECG signal file with precise time stamps for offline analysis. Therefore, the novel system is able to provide real-time VA monitoring and can be used to analyze the stored ECG retrospectively for any type of arrhythmia event and VA. In addition to ECG monitoring, the novel system processes S1S1 and S1S2 stimulating programs with several adjustable parameters. The continuous stimulation of IECD operates for at least three months. VAs were readily induced (75%) in rabbits with MI, and then terminated (94%) in rabbits pre- and post-MI surgery using the multifunctional simulation system. The novel system with high-quality ECG signals and advanced stimulation functionality can be used to study the management of VAs in awake and active animals without the requirement of anesthetics for acute and chronic studies. Thus, the system may be useful for experimental studies in terms of VAs in heart failure, and for exploring the efficacy of novel drugs and testing the feasibilities of using novel devices to manage VAs (14).

Telemedicine is one of the most attractive areas of modern medicine (15). Thus far, there have been relatively few research studies concerning the role of web-based remote management of VAs, in contrast to the wealth of studies on internet interventions to support the remote management of other conditions (16,17). If it is possible to use the web-based remote rescue method to save the lives of patients with malignant VAs in the future, the mortality rate due to cardiovascular events and SCD is likely to be reduced significantly.

Therefore, the final goal of the new system is to develop a novel remote clinical medical device for patients with heart disease and arrhythmias. This novel system may be used for round-the-clock real-time wireless ECG monitoring of patients with VAs or with high risk of VAs, with unexplained syncope or palpitations with possible arrhythmic origin, or to measure the burden of atrial fibrillation, similarly to other types of implantable subcutaneous cardiac monitors (6). In addition to the ECG monitoring function, the ATP function is another method of managing VAs with this system. Numerous clinical studies have shown that the majority of VA events resulting from VT are terminated by ventricular pacing (11,12,18,19). In the present study, induced VAs were effectively terminated by ATP in the rabbit model. The novel equipment may be used to monitor and terminate VAs in patients at high risk in the future.

However, extensive improvements and further study are required in order to achieve the clinical use of this device. Presently, the novel equipment described in the present study is under development and a number of drawbacks remain to be overcome. The current system does not provide a defibrillator function. As VF may be triggered by the ventricular simulation, it would be better and safer to combine the defibrillator function in the implanted system. In addition, only one pair of electrodes was used in the present study. A single ECG monitoring channel occasionally limits the diagnostic capability. Furthermore, beat-to-beat manual ECG analysis is a time-consuming process (20,21) and this system requires integration of an automatic analysis system. The model switch with a wireless signal transceiver, a signal transfer device of the extracorporeal system, should be miniaturized to the size of a mobile phone to enable it to be easily carried by the patient. Also, internet safety must be guaranteed to prevent hacker manipulation on the stimulation system and ensure the safety of patients.

In conclusion, the web-based newborn IECD system with a real-time remote ECG monitoring and stimulation system supplies a useful method of creating an animal model, which may be used in acute and chronic experimental studies concerning the development of novel drugs and devices for the management of VAs. Extensive future studies are required to develop novel versions of the IECD system, which may enable the diagnosis and termination of VAs.

## Figures and Tables

**Figure 1:** External features and components of the implantable electronic cardiovascular device. ECG, electrocardiogram.

**Figure 2:** Schematic diagram of the implantable electronic cardiovascular device (IECD) implanted in a rabbit and the extracorporeal remote system. 3G, third-generation mobile communications technology.

**Figure 3:** ECG signaling was recorded synchronously by surface (upper) and remote (lower) ECGs. (A) Normal sinus rhythm; (B) ventricular pacing; (C) VF; and (D) VT. ECG, electrocardiogram; VF, ventricular fibrillation; VT, ventricular tachycardia.

**Figure 4:** S1S1 (upper) and S1S2 (lower) programs. S1S1, regular stimuli; S1S2, regular stimuli with an added early-extra-stimulus.

**Figure 5:** Correlation between the stimulating current and the stimulating signal voltage recorded by the surface and remote ECGs (upper graphs). Correlation of the stimulating signal voltage between the remote and surface ECGs (lower graph). ECG, electrocardiogram.

**Figure 6:** VT induced and then terminated by the S1S2 pacing program (upper graphs). VT/VF induced and then terminated by the S1S2 pacing program (lower graphs). SR, sinus rhythm; VT, ventricular tachycardia; VF, ventricular fibrillation; S1S2, regular stimuli with an added extra stimulus.

## Abbreviations

VA: ventricular arrhythmia
VT: ventricular tachycardia
VF: ventricular fibrillation
IECD: implantable electronic cardiovascular device
MI: myocardial infarction
S1S1: regular stimuli
S1S2: regular stimuli with an added extra stimulus
SCD: sudden cardiac death
ATP: anti-tachycardia pacing
